# Teledentistry as a Supportive Tool for Dentists in Diagnosing MRONJ in Northern Cyprus

**DOI:** 10.1155/2021/5657152

**Published:** 2021-12-29

**Authors:** Mujgan Firincioglulari, Kaan Orhan

**Affiliations:** ^1^Final International University, Faculty of Dentistry, Department of Dentomaxillofacial Radiology, Nicosia, Cyprus; ^2^Ankara University, Faculty of Dentistry, Department of Dentomaxillofacial Radiology, Ankara, Turkey; ^3^Ankara University Medical Design Application and Research Center (MEDITAM), Ankara, Turkey; ^4^Department of Dental and Maxillofacial Radiodiagnostics, Medical University of Lublin, Poland

## Abstract

**Objective:**

This web-based survey, as a tool of teledentistry, is aimed at assessing the level of knowledge, attitudes, and awareness regarding MRONJ among dental professionals in Northern Cyprus.

**Methods:**

An online self-administered questionnaire about MRONJ was sent to all dentists in Northern Cyprus through Google Forms. The first part of the questionnaire consists of demographic and professional information, and the second part included questions about knowledge and awareness questions about MRONJ. The SPSS software was used for statistical data analysis. A Chi-square test was performed to compare between the groups. The significance level was set at *p* < 0.05.

**Results:**

A total of 112 dentists participated in this survey. The participants showed an insufficient level of knowledge regarding MRONJ, as only 56.6% of the participants stated that they had general knowledge about MRONJ. Regarding the practical questions of the survey, the participants showed poor knowledge about implant and tooth extraction procedures while a patient is using antiresorptive or antiangiogenic drugs, particularly the usage of oral antiresorptive or antiangiogenic drugs for less than 3 years. Participants showed adequate knowledge in terms of usage area of medications and administration of them.

**Conclusion:**

Teledentistry can be used as a supportive tool for dentists in diagnosing MRONJ. Similar to previous studies, the knowledge and awareness of MRONJ of dentists in Northern Cyprus were found to be inadequate. There is a significant need to provide more professional information as part of undergraduate programs so that the next generation of dentists can practice more confidently.

## 1. Introduction

Teledentistry is the use of health information about health technology and telecommunications for oral healthcare, education, consultation, and public knowledge to improve oral health [1].

Teledentistry is the remote facilitating of oral care, education, and guidance as a substitute to direct face-to-face contact with any patient or colleague. After years, teledentistry has been validated to be useful for a remote dental screening, providing consultation, making the diagnosis. Teledentistry is found to be comparable to real-time guidance in rural areas with limited access to facilities and long-term healthcare facilities. It makes use of Information and Communication Technology (ICT), especially of the Internet, to transfer clinical information [2, 3].

ICT used in partnership with the Internet has become an important element of academic life in universities. Internet-based teledentistry education permits people to choose the time, place, and type of education [4]. As with many parts of telemedicine, teledentistry usage has been steadily increasing. Telehealth has been supported by many institutions to perform a critical role in preserving communication with patients [5].

In today's circumstances of continuing the COVID-19 pandemic, the essential goal is to avoid person-to-person contact because it spreads by droplet, fomite, and contact transmission. The word “tele” means “distant,” and thus, teledentistry provides the need for social distancing as has been advocated by health authorities all across the world to stop the spread of the SARS-COV-2 virus [2].

Medication-related osteonecrosis of the jaw (MRONJ) is a common serious side effect of using antiresorptive (AR) (bisphosphonates (BP) or denosumab) or antiangiogenic (AA) drugs. These drugs are used in the treatment of hypercalcemia and bone metastases in cancer patients (e.g., multiple myeloma) or to prevent fragility fractures in osteoporosis patients [6].

MRONJ can be considered if the following situations are present: the use of antiresorptive or antiangiogenic agents for current or previous treatment, exposed bone or bone that can be probed through a fistula in the maxillofacial region for at least 8 weeks, and no history of head and neck radiation therapy [7].

Antiresorptive (BP or denosumab) drugs reduce the resorption of bone, pain, and fracture risk in patients with bone disease. On the other hand, antiangiogenic drugs affect angiogenesis which impedes healing. These medications alter bone remodeling by connecting to mineralized bone tissue and by the adverse impact on osteoclast function [8]. In 2003, it was first accepted that bisphosphonate-related osteonecrosis of the jaw is a side effect for patients who are using intravenous bisphosphonates as treatment of malignant diseases with bone metastases [9]. The duration and type of treatment, as well as medical anamnesis, could affect the risks for the patients [10].

The epidemiology and pathogenesis of MRONJ are still unknown; however, a growing body of evidence indicates that MRONJ is a multifactorial process associated with retarded epithelial regeneration, diminished vascularity, and failure of bone remodeling processes. Several risk factors have been stated, including duration of used medications, route of administration (for example, the risk is significantly higher with intravenous medications), dentoalveolar surgery, age, and systemic diseases. Moreover, remarkable development has been achieved in terms of the prevention of MRONJ by studying local risk factors such as the presence of inflammatory, dental-periodontal, and/or peri-implant diseases [11–13]. Figures 1 and 2 show the intraoral and radiological appearance of MRONJ.

MRONJ can be classified and staged with a system proposed by The American Association of Oral and Maxillofacial Surgeons (AAOMS) in 2014, which has been generally used since that time [14].

Dentists have an important role in the prevention and early diagnosis of MRONJ. The treatment can be difficult and can lead to serious types of pain and lessened quality of life. Many studies have shown that preventive oral hygiene procedures incorporated with effective dental health practices are correlated with a lower rate of MRONJ. In light of this situation, the American Society of Clinical Oncology and Cancer Care Ontario made the following suggestion: “A dental evaluation is recommended, where appropriate, before initiation of bisphosphonates, and any pending health or oral problems should be dealt with before starting treatment [14, 15]. Therefore, dental practitioners must have sufficient knowledge of MRONJ, its potential complications, and treatment planning in patients at risk of MRONJ [13].

Recent researches from dentists around the whole world reveal that most of these participants have inadequate knowledge about MRONJ as an adverse effect of these drugs [10, 13, 16–20]. Awareness and knowledge about MRONJ are essential for all dentists to diagnose “at at risk” patients for suitable consultation and management [17].

In diagnostic dentistry, it can be challenging to diagnose oral lesions accurately, especially in rural communities with limited access to specialized dental care. Thus, teledentistry may fill this gap and develop the standard of oral care [21].

With the number of patients on bisphosphonates and other antiresorptive drugs increasing, dental practitioners can play an important role in the prevention of MRONJ in patients receiving bisphosphonate therapy, and there are no previous survey reports about dentists' knowledge concerning bisphosphonate therapy in North Cyprus.

Therefore, this cross-sectional web-based survey, as a tool of teledentistry, is aimed at assessing the level of knowledge and awareness among dental professionals in Northern Cyprus regarding MRONJ.

## 2. Materials and Methods

This descriptive cross-sectional study was performed using Google Forms, and the link was sent through e-mails or WhatsApp groups to all dentists in Northern Cyprus from March to May 2021. The survey study is designed to assess the awareness, knowledge, management, and practice of all dentists concerning MRONJ patients. The inclusion criteria of the study were being a dental specialist or general dentist. The exclusion criteria of the survey were being a dental student or intern. A cover letter explaining the aim of the survey and identifying the research team was also included in the web form. The study was approved by the Research and Ethics committee (IRB Number: 24/21) conforming to the 1964 Helsinki Declaration and its later amendments or comparable ethical standards. The participants were made aware of the study aim, the importance of the survey, and the researcher's name. To ensure confidentiality, the participants were informed that their names were not required on the questionnaire.

The multiple-choice questionnaire was sent to 160 dentists, out of which 112 responses were obtained. The self-administered questionnaire was modified from previously corroborated questionnaires that had been used in similar reports [13, 16–18, 20]. When the participants had any questions, they were answered by e-mail, and they were asked to mark their answers and complete them by themselves.

This questionnaire consists of two main parts. The first section consists of 4 demographic and professional questions including gender, age, years of experience (1-10, 10-20, or >20), and specialization (general dentist or specialist). The second part consists of 18 knowledge and awareness questions about MRONJ (commercial names, therapeutic indications of medication, route of administration and risk factors, and clinical features of MRONJ and questions like case study).

### 2.1. Statistical Analysis

Responses obtained from this survey study were performed descriptively. All responses were presented in the form of frequencies and percentages. Comparisons were made by using the chi-square test. All statistical analyses were performed with SPSS for Windows version 15.0 (SPSS Inc., Chicago, IL). The significance level was set at *p* < 0.05.

## 3. Results

### 3.1. Demographic Information

A questionnaire link was sent to a total of 160 dentists in Northern Cyprus, out of which 112 dentists responded. 64% of the participants were female, and 36% were male. The mean age of the participants was 32.2 (range 23-66). Participants were categorized according to specialization where 46.5% of the participants were general dentists and the rest of the participants had a postgraduate degree, specialized in either Dentomaxillofacial Radiology, Dentomaxillofacial Surgery, Periodontology, Orthodontics, Pedodontics, Endodontics, Restorative Dentistry, or Prosthodontics. 78.9% of the participating dentists had between 1 and 10 years of experience.  Table 1 shows the detailed demographic and characteristic information of the participants.

### 3.2. Knowledge and Awareness of Participants

56.6% of the participants stated that they had general knowledge about MRONJ, and 11.5% stated that they did not know, while 31.9% indicated that they were not sure about their knowledge. According to the area of specialty in orthodontics, pedodontics, and restorative specialties, less than 35% of the participants in each specialization stated that they knew MRONJ. 52.4% of the specialists and 47.6% of the general dentists expressed that they knew MRONJ. The relationship between knowledge about MRONJ and the area of specialty can be seen in Table 2. There was no significant relationship between general knowledge about MRONJ and years of practice (*p* > 0.05).

The participants were asked about the usage area of AR and AA drugs; the results showed that osteoporosis was the most stated answer with the rate of 83.2%, followed by bone metastasis (73.5%), multiple myeloma (39.8%), osteogenesis imperfecta (23.9%), and anemia (0.9%) (Figure 3). According to the area of specialty, the results showed that only 2 participants (1 general dentist and 1 oral surgeon) stated anemia for bisphosphonate usage, whereas more than 70% of the participants in every specialty answered osteoporosis except pedodontics. Bone metastasis and osteogenesis imperfecta are considered as an answer in every specialty area almost equally except general dentists, orthodontics, and endodontics. These three specialties showed lower percentages. Osteoporosis and bone metastasis showed almost equal percentages of answers in the range of years of experience. On the other hand, multiple myeloma and osteogenesis imperfecta showed lower percentages in dentists with more than 20 years of experience.

Fosamax (73%) and Zometa (61%) had the highest percentage for the question regarding medications that can produce osteonecrosis.  Figure 4 shows the details of the answers for medications that can produce osteonecrosis.

The results were compared with years of experience, and no significant difference was found between the answers and years of experience. In addition, answers were compared between general dentists and specialists, and the results showed that there was a significant difference in terms of the answers regarding Actonel and Bonviva between general dentists and specialists (*p* < 0.05). Specialists stated that Actonel and Bonviva are medications that can produce osteonecrosis more than general dentists (Table 3).

93% and 78.1% of the participants expressed that AR and AA drugs can be administered orally and intravenously, respectively (Figure 5). There was no significant difference according to the area of specialty. On the other hand, in terms of years of experience, a significantly higher proportion of dentists with 1-10 years of experience selected IV as an answer (86.5%) compared with dentists who had 10-20 years (44.4%) and <20 years of experience (54.5%) (*p* < 0.05) (Table 3). Only 25.9% of the participants indicated that they were familiar with at least one guideline for MRONJ treatment. 73.2% of the participants responded posterior mandibular to this question, followed by the anterior mandibula (17%), posterior maxilla (6.3%), and anterior maxilla (3.6%). There was no significant difference between years of experience and areas of specialty. 84.4% of the participants stated that patients with IV AR and AA drug usage had a greater prevalence of MRONJ than oral users (15.6%). All specialties except pedodontics selected IV administration as the answer with a rate of more than 84%. Only 55.6% of the pedodontics specialty participants chose IV as their answer.

61.4% of the participants agreed with the phrase of good oral hygiene reduces the risk of MRONJ while 22.8% said that they were not sure, and 15.8% of the dentists disagreed with oral hygiene and the MRONJ relationship. The percentage of “not sure” answers increased in line with the number of years of experience.

### 3.3. Practical Questions (Table 4 Shows the Detailed Results)

About the question about tooth extraction:

- *Taking AR and AA Drugs Intravenously before the Tooth Extraction Procedure*. 36.8% stated that they would suspend the bisphosphonate treatment for 3 months and then proceed with the treatment, whereas 30.7% stated that would administer no treatment, 27.2% stated they were not sure, and 5.3% indicated that they would carry out the treatment
- *Using AR and AA Drugs Orally for Less than 3 Years*. 45.3% stated that they would suspend the bisphosphonate treatment for 3 months, and 29.5% said they were not sure, while the results for no treatment and carry out the treatment were the same (12.6%)
- *Orally for More than 3 Years*. 41.2% stated that they would suspend the AR and AA drug treatment for 3 months, 28.1% said they would apply no treatment, 24.6% were not sure, and 6.1% stated that they would carry out the treatment

Regarding the question about implants:

- *Taking AR and AA Drugs Intravenously before Implant Replacement*. 45.6% of the participants stated no treatment as their answer, 28.1% stated that they were not sure, 24.6% said they would suspend the AR and AA drugs treatment for 3 months and then proceed with the treatment, and 1.8% responded that they would carry out the treatment
- *Using AR and AA Drugs Orally for Less than 3 Years*. 32.6% of the participants were not sure about this question, 29.5% stated no treatment, 28.4% said they would suspend the AR and AA drugs treatment for 3 months and then proceed with the treatment, and finally, 9.5% said they would carry out the treatment
- *Orally for More than 3 Years*. 41.2% stated that they would suspend the AR and AA drug treatment for 3 months, 28.1% stated no treatment, 24.6% were not sure, and 6.1% responded that they would carry out the treatment

## 4. Discussion

The theory of teledentistry was initially introduced by the American Army as part of the Total Dental Access Project in 1994. The main aim was to increase the productivity of dental services delivered to soldiers. Currently, teledentistry is commonly accepted in the fields of dental education, public awareness, and research activities [1, 21].

Through advancing technology, there has been a radical adjustment in offering oral health care to patients. One such modification is because of the budding field of teledentistry. It can be of different types such as patient–dentist, dentist–specialist, dentist–data storage bank, students–dental education, and dentist–research center [22].

The application of teledentistry in oral medicine and diagnosis was evaluated through research performed in Northern Ireland, where the authors used a prototype teledentistry system as part of a service advancement scheme and the authors expressed that teledentistry may serve as an alternative way to administer referrals in oral medicine [23].

Diagnosis of oral lesions could be discussed via teleconsultation, which is contributing to a greater resolution of clinical cases. The challenging diagnosis of oral lesions is one of the reasons for the delayed diagnosis of malignant lesions [24].

The advantages of the web-based self-administered survey are appealing to surveyors because they allow for rapid improvement and administration of surveys, low cost, fast data collection, and analysis. Internet surveys may be suggested for the use of clinical and academic research settings with improved speed and effectiveness of data collection compared with verbal or paper survey methods [25].

On the other hand, comparatively high nonresponse rates than traditional methods of data collection and concerns regarding the reliability and validity of the data obtained could be disadvantages of a web-based survey. Additionally, participants could be hesitant to use web-based surveys because safety and confidentiality issues may also play a role [26].

In this manner, a web-based survey as a tool of teledentistry helps in the diagnosis of MRONJ by providing communication between dentists.

MRONJ is more common in cancer patients (1.8–5% incidence) than osteoporosis patients (0.01–0.03% incidence); this is partly due to the medical condition, but also the doses and potency of AR or AA drugs used. It can lead to debilitating effects due to unexplained causes [27, 28]. The first series of cases of osteonecrosis of the jaw related to medications were reported by Marx at the University of Miami in 2003 and involved 36 cases of painful bony exposure in the maxilla and mandible that were not responding to any surgical or medical treatment in patients receiving intravenous bisphosphonates [29]. Globally, the percentage of people aged older than 65 years has increased because of a lengthened average lifetime [30]. Therefore, this has led to an increase in the number of patients with osteoporosis, which increases the use of antiresorptive drugs, heightening the risk of an increased number of MRONJ cases [31]. The increase in the incidence of MRONJ highlights the importance of the knowledge and awareness of dentists about MRONJ. This study surveyed dentists in Northern Cyprus to evaluate their awareness, knowledge, and risk factors regarding MRONJ.

The results of this evaluation were concerned in terms of the knowledge on MRONJ among the participant dentists. There was no significant difference concerning the level of knowledge among respondents with higher degrees (specialists) compared with general dentists.

The responses to the first and basic question of the questionnaire, which was about the knowledge of MRONJ, indicated that just 56.6% of the participants had heard about the disease and the majority of participants could not recognize the commercial names of antiresorptive or antiangiogenic drugs. This was evidence of poor knowledge of MRONJ among the surveyed dentists. Previous studies have also reported very poor knowledge on MRONJ among dentists, as in our study [13, 16–18, 20, 32]. Rosella et al. [33] suggested that greater educational efforts should be implemented regarding MRONJ in undergraduate degree programs. Thus, the results of our study and similar researches could be attributed to insufficient education about MRONJ at the undergraduate level.

MRONJ negatively affects the life quality of patients, which can lead to morbidity in affected patients. Thus, dentists should not only have sufficient knowledge and awareness about MRONJ but also adequate knowledge regarding the suitable treatment strategies in patients undergoing antiresorptive or antiangiogenic drug therapy. Fortunately, AAOMS has established very distinct guidelines regarding MRONJ staging and treatment planning of patients at risk of this eviscerating disease. However, only 25.9% of the participating dentists were familiar with the guidelines, which is a similar finding to several studies that reported that the majority of dentists were not familiar with any guidelines [18, 20, 34].

Escobedo et al. [20] and Al-Hussain et al. [35] reported that knowledge of MRONJ treatment and management decreases with years of experience, especially among professionals with more than 20 years of experience. Similarly, de Lima et al. [36] found that participants with less than 5 years of experience had the highest scores for the risk factors related to the development of MRONJ. On the other hand, Miranda-Silva et al. [32] reported that the MRONJ knowledge scores tended to increase with years of experience. In our study, there were only significant differences according to years of experience in the administration of antiresorptive or antiangiogenic drugs and treatment strategies in tooth extraction while the patient was using BPs. The results showed that for these two questions, dentists with 1-10 years of experience had significantly better knowledge. For other questions, there was no significant difference according to years of experience.

In previously reported studies, in the evaluation of knowledge regarding the therapeutic indications for bisphosphonates, antiresorptive, or antiangiogenetic, osteoporosis was the most stated answer by participants followed by cancer treatment for bone metastases and multiple myeloma and osteogenesis imperfecta [13, 33, 34, 37]. These previous reports verify the results of this survey that osteoporosis was the main therapeutic indication stated by the dentists, followed by cancer treatment of patients with metastatic bone tumors, multiple myeloma, and osteogenesis imperfecta and anemia.

Al-Hussain et al. [35] reported a survey conducted with general dentists and specialists. Based on the results, it was concluded that participants were precautious about performing oral surgery on patients taking BPs. In that study, participants who achieved higher scores in knowledge recommended that greater educational information should be given to dentists regarding MRONJ complications. Our study results also support this outcome. More educational material about MRONJ should be provided to undergraduate students. The prevention of MRONJ requires more information than just adequate awareness and knowledge on MRONJ. It is a reality that patients have insufficient knowledge about the drugs they are using.

Communication between professionals is essential for MRONJ patients and their quality of life; communication must become routine to enhance patient care and correctly handle patients at risk of developing MRONJ.

There were several limitations in the present survey. Firstly, the number of participants was relatively low due to the small community of dentists in Northern Cyprus. Moreover, 78.9% of participants had between 1 and 10 years of experience. Only 16 of the dentists who participated in the survey had more than 20 years of experience. The lack of experienced participants had a significant impact on the outcomes of this study. Furthermore, this was a self-administered questionnaire so the responses may not have revealed the actual knowledge of the participating dentists. Despite these limitations, we believe that this survey has provided helpful information on the level of MRONJ awareness and knowledge among dentists around the world.

## 5. Conclusion

Teledentistry can be used as a supportive tool for dentists in diagnosing MRONJ. Similar to previous studies in other countries, the knowledge and awareness of MRONJ among dentists practicing in Northern Cyprus were found to be inadequate. Such alarming results demonstrate that more professional information must be given in undergraduate programs so that the next generation of dentists can practice more confidently and effectively with MRONJ patients. Moreover, experienced dentists should refresh their knowledge with seminars and educational programs.

## Figures and Tables

**Figure 1:** Panoramic and cone beam computed tomography images of MRONJ.

**Figure 2:** Intraoral image of MRONJ.

**Figure 3:** Percentage of participants' answers related to the usage area of bisphosphonates.

**Figure 4:** Percentage of participants' answers related to medications that can produce osteonecrosis.

**Figure 5:** Percentage of participants' answers to the administration of AR and AA drugs.

**Table 1:** The detailed demographic and characteristic information of participants.

	Frequency	Percent (%)
Gender		
Male	41	36
Female	73	64
Area of speciality		
General dentistry	53	46.5
Dentomaxillofacial Radiology	2	1.8
Dentomaxillofacial Surgery	10	8.8
Periodontology	8	7
Endodontics	6	5.3
Prosthodontics	13	11.4
Orthodontics	5	4.4
Pedodontics	10	8.8
Restorative Dentistry	7	6.1
Years of experience		
1-10 years	90	78.9
10-20 years	8	7
>20 years	16	14

**Table 2:** Knowledge about MRONJ according to the specialties.

			Specialty									Total
			General dentist	Dentomaxillofacial Surgery	Orthodontics	Periodontology	Endodontics	Prosthodontics	Pedodontics	Dentomaxillofacial Radiology	Restorative Dentistry	
									
Knowledge about MRONJ	Yes	*N*	30	9	1	5	4	7	3	2	2	63
		% within speciality	56.60%	100.00%	20.00%	62.50%	66.70%	53.80%	30.00%	100.00%	33.30%	56.30%
	No	*N*	4	0	2	0	1	1	3	0	2	13
		% within speciality	7.50%	0.00%	40.00%	0.00%	16.70%	7.70%	30.00%	0.00%	33.30%	11.60%
	Not sure	*N*	19	0	2	3	1	5	4	0	2	36
		% within speciality	35.80%	0.00%	40.00%	37.50%	16.70%	38.50%	40.00%	0.00%	33.30%	32.10%
Total		*N*	53	9	5	8	6	13	10	2	6	112
		% within speciality	100.00%	100.00%	100.00%	100.00%	100.00%	100.00%	100.00%	100.00%	100.00%	100.00%

**Table 3:** Knowledge of different AR and AA drugs by participants and comparison of administration of bisphosphonates with years of experience. Italic shows statistical significance (*p* < 0.05).

Medication	Dentists (%)	Specialists (%)	*p* value		Years of experience			
Alendronate (Fosamax ©)	56.6%	71%	*p* > 0.05	Administration	1-10	10-20	>20	*p* value
Zoledronic acid (Zometa ©)	50.9%	53.3%	*p* > 0.05	Intravenously	86.5%	44.4%	54.5%	*p* = 0.001
Risedronate (Actonel ©)	5.7%	25.0%	*p* = 0.009^∗^	Intramuscularly	10.1%	0	18.2%	*p* > 0.05
Ibandronate (Bonviva ©)	17%	38.3%	*p* = 0.013^∗^	Oral	91%	100%	100%	*p* > 0.05
Denosumab (Prolia ©)	17	16.7%	*p* > 0.05	Subcutaneously	1.1%	11.1%	0	*p* > 0.05

**Table 4:** Guideline for tooth extraction and implants in patients with BP treatment and percentage of right answers among general dentists and postgraduate dentists with years of experience.

	IV AR and AA drugs	Oral AR and AA drugs < 3 years	ORAL AR and AA drugs > 3 years
Tooth extraction	Right answer: no treatment	Right answer: carry out treatment	Right answer: suspend AR and AA drugs for 3 months
	General dentists: 28.3%	General dentists: 14.3%	General dentists: 39.6%
	Specialists: 31.7%	Specialists: 12.1%	Specialists: 40%
	*p* > 0.05	*p* > 0.05	*p* > 0.05
	1-10 years exp. = 34.8%	1-10 years exp. = 10.8%	1-10 years exp. = 41.6%
	10-20 years = 0%	10-20 years = 33.3%	10-20 years = 33.3%
	>20 years = 9.1%	>20 years = 18.2%	>20 years = 45.5%
	*p* < 0.05^∗^	*p* > 0.05	*p* > 0.05
Implants	Right answer: no treatment	Right answer: carry out treatment	Right answer: suspend AR and AA drugs for 3 months
	General dentists: 41.5%	General dentists: 8%	General dentists: 39.6%
	Specialists: 43.3%	Specialists: 11.9%	Specialists: 26.7%
	*p* > 0.05	*p* > 0.05	*p* > 0.05
	1-10 years exp. = 40.4%	1-10 years exp. = 8.2%	1-10 years exp. = 32.6%
	10-20 years = 33.3%	10-20 years = 33%	10-20 years = 44.4%
	>20 years = 54.5%	>20 years = 9.1%	>20 years = 27.3%
	*p* > 0.05	*p* > 0.05	*p* > 0.05

## Data Availability

The datasets used and/or analyzed during the current study are available from the corresponding author on reasonable request.
